# Sports Augmented Cognitive Benefits: An fMRI Study of Executive Function with Go/NoGo Task

This article has been retracted.

**DOI:** 10.1155/2021/7476717

**Published:** 2021-12-07

**Authors:** Qingguo Ding, Lina Huang, Jie Chen, Farzaneh Dehghani, Juan Du, Yingli Li, Qin Li, Hongqiang Zhang, Zhen Qian, Wenbin Shen, Xiaowei Yin, Pei Liang

**Affiliations:** ^1^Imaging Department, Changshu No. 2 People's Hospital (The Clinical Medical College Affiliated to Xuzhou Medical University), Changshu, China; ^2^Department of Psychology, Faculty of Education, Hubei University, Wuhan, China; ^3^Department of Psychiatry, Research Center of Addiction and Behavioral Sciences, Shahid Sadoughi University of Medical Sciences, Yazd, Iran; ^4^The School of Education, Soochow University, Soochow, China; ^5^Brain and Cognition Research Center, Faculty of Education, Hubei University, Wuhan, China

## Abstract

Exercise is believed to have significant cognitive benefits. Although an array of experimental paradigms have been employed to test the cognitive effects on exercising individuals, the mechanism as to how exercise induces cognitive benefits in the brain remains unclear. This study explores the effect of dynamic neural network processing with the classic Go/NoGo task with regular exercisers. We used functional magnetic resonance imaging to analyze the brain activation of areas involved in executive function, especially inhibitory control. Nineteen regular joggers and twenty-one subjects as a control group performed the task, and their brain imaging data were analyzed. The results showed that at the attentive visual period, the frontal and parietal areas, including the prefrontal cortex, putamen, thalamus, lingual, fusiform, and caudate, were significantly enhanced in positive activities than the control group. On the other hand, in the following inhibitory control processing period, almost the same areas of the brains of the exercise group have shown stronger negative activation in comparison to the control group. Such dynamic temporal response patterns indicate that sports augment cognitive benefits; i.e., regular jogging increases the brain's visual attention and inhibitory control capacities.

## 1. Introduction

Exercise is getting increasingly popular, and it has become one of the significant designators to indicate one's social status. Different studies have evidenced that exercise can shape the brain structure and lead to cognitive benefits. Variant cognitive task paradigms have been applied to explore the relationship between exercise and the brain's cognitive function, such as executive function [1], attention [2], and memory [3]. The elderly subjects with higher aerobic exercise have the greater gray matter capacity of the prefrontal cortex and larger gray matter volume, such as the dorsolateral prefrontal cortex (DLPFC) [4]. They improved attention and memory and performed better in the Stroop and Spatial Working Memory (SPWM) tasks. Exercise training can increase the individual's exercise adaptability and improve cognitive performance, especially in perception speed and executive control [5]. Independent of ages, a similar performance effect has been observed in the adult population for the enhanced inhibition control and the reevaluation of cognitive ability [6].

How is the processing of exercise shaping the brain? It is essential and urgent to understand the etiology of the brain mechanism involved in the exercise-induced neural process of functional cognitive benefits. The cue reactivity and inhibitory control are the critical processes involved in developing and maintaining motion ability and capacity. Traditionally, the Go/NoGo (GNG) task has been used as a tool to observe the inhibition function in the brain network processing by comparing the Go and the NoGo conditions. For instance, an electrophysiological (EEG) study showed that elite athletes performed GNG tasks better than the table tennis college students [7]. The authors observed a pronounced “NoGo effect” of the larger N2 and P3 components with the athletes, indicating a more substantial inhibitory function [7]. Although the EEG data has a very rough spatial resolution, the electrodes recorded from the frontal-central and central-top areas have shown stronger athletes' responses than those of the college students, under the conditions of Go and No Go. Similarly, the GNG [8] and Stroop Color Word (SCW) tasks [9] both elicit the negative amplitudes of N200 and N450 with a frontal/frontocentral distribution and in the anterior cingulate cortex [10, 11]. A positive-going amplitude of P300, peaks at parietal/centroparietal regions, was observed [12, 13]. The magnitude of P300 is suggested to be proportional to the allocation of attentional resources to evaluate task-relevant stimuli [14]. The task-relevant stimuli may activate the shared set of the neural network, including attention, inhibitory control, and other cognitive-related function. The exerciser could perceive task cues and evoke better attentive behavior. They perform the task better, especially with the inhibitory behavior such as the NoGo task. However, the brain mechanism of exercise above-mentioned was mostly discovered with EEG recordings. The complex neural networks involved with enhanced cue reactivity and response inhibition remain unclear. Hence, it is urgent to look exactly into the complex neural networks of the particular cognitive benefits. Functional magnetic resonance imaging (fMRI) can help to locate the brain activities in detail. Therefore, in this study, we aim to observe the neural response patterns of habituated exercisers with fMRI. In doing so, the effect on dynamic neural network processing with the classic GNG task with regular exercisers will be analyzed. The results will also be compared with the previous literature.

In order to delineate the mechanism of exercise-induced visual cue responses and inhibitory responses, we hypothesized the following: (1) visual cue responses would be enhanced. In other words, the exercise group would demonstrate increased cue reactivity in mesolimbic dopamine regions in the presence of cues; (2) inhibitory systems would be enhanced. There would be stronger negative responses of prefrontal neural activity during response inhibition compared to controls. In the end, by testing our hypothesis with the observed neural correlates, we could compare the results with other exercise behavioral studies and discuss the validity of exercise shaping cognitive benefits.

## 2. Methods and Materials

### 2.1. Participants

The free volunteers were selected through a social media advertisement, precisely on WeChat, which lasted for about three months in Changshu, China. The participants of the exercise group were mainly members of the local running clubs in Changshu. The total number of subjects in the exercise group was 19, including 13 males and 6 females (average age: 45.42 ± 3.50 years). As a control group, 21 nonathletic enthusiasts were recruited, including 10 males and 11 females (average age: 46.10 ± 5.16 years). No significant difference was observed in the gender (chi-square, *p* = 0.184), age, and education years (*t*-test, both *p* > 0.05) among the subjects of the exercise group and the control group. All subjects reported normal or corrected vision and no history of mental disorder problems.

All the volunteers had regular office sedentary work, and none of them was a full-time or part-time athlete. We selected the participant as the exercise group (1) if she/he had participated in a marathon at least once a month, (2) if she/he had jogging at least three times a week, and (3) if each of their jogging sessions lasted more than one hour. The frequencies, the total exercise time per week, and the control groups are compared and listed in Table 1. After comparing the columns of Table 1, it can be seen that the frequencies and the total exercise time per week of the exercise group are significantly higher than those of the control group.

All the subjects were well informed about the procedures of this study and before the experiment were made to sign the written consent. The study was approved by the Ethics Committee (IEC) of the No. 2 People's Hospital of Changshu (license number 2018-68), according to the Ethics Guidelines.

### 2.2. Tasks

After the participants were recruited and selected, they were scheduled to be scanned for the GNG tasks. The participants executed the traditional GNG task with an event-related design. The stimuli contained 26 black capital alphabets on the white background of the display. On display, the stimuli are divided into two groups: X group with 20% frequency and non-X group with 80% frequency. Each trial began with a fixation (+) on display for 750 ms, followed by an alphabet presented for 250 ms. Then, the black screen lasted for 1000 ms. During the presentation of the black screen, the participants were requested to identify the alphabet and press the button with the right hand if the alphabet was non-X (the Go trial) or not respond at all, if it was X (the No Go trial). The block consisted of 120 trials, and after 1 min break, the block was to be repeated once more. The whole run lasted around 9 min.

### 2.3. MRI Data Acquisition

Structural and functional MRI data were collected using the GE Discovery MR750W 3.0 T scanning system, housed in the Imaging Department of No. 2 People's Hospital of Changshu. The scanner was with the 8-channel head coil. During the scanning process, the participants were quietly lying on the back in the magnetic resonance examination bed, fixing the head inside the head coil with foam padding, and wearing earplugs to reduce machine noise. The participants watched the visual stimuli through a reflector mirror mounted on the head coil. Through the mirror, the visual stimuli were reflected from the projector screen, placed outside the gate of the MRI. For structural imaging, high-resolution T1-weighted scans were acquired. The 3D T1 BRAVO_SPM volume sequence was applied with TR = 8.5 ms, TE = 3.2 ms, flip angle = 12°, FOV = 24 cm, 256 × 256 matrix size, and 1 mm slice thickness. The MR sequence for T2-weighted functional imaging was acquired using TR = 2000 ms, TE = 30 ms, flip angle = 90°, scan resolution of 64 × 64, 33 slices, intervals of 0.2 mm with slice thickness = 3.6 mm, FOV = 24 cm, and voxel size = 3.75 × 3.75 × 3.75 mm^3^. The first 2 scans were discarded to allow for the BOLD signal to stabilize.

### 2.4. fMRI Data Analysis

Preprocessing and statistical analysis of fMRI data were performed using SPM12 (Wellcome Department of Imaging Neuroscience, University College London, UK, http://www.fil.ion.ucl.ac.uk/spm), implemented in MATLAB R2013b (MathWorks, Inc., Natick, MA). The preprocessing included head motion correction, spatial normalization, and spatial smoothing with a 6 mm full-width at half-maximum Gaussian kernel. The coregistered functional and anatomical images were registered to Montreal Neurological Institute (MNI) space, with a resolution of 3 × 3 × 3 mm^3^. The sequences with head movement range exceeding 3 mm or rotation that exceeded 3 degrees were removed.

After the preprocessing was completed in a first-order analysis, the evoked hemodynamic responses under three conditions were modeled for each subject, using box-car functions to convolve with canonical HRF (hemodynamic response function) to construct a general linear model (GLM). The nuisance regressor consisted of the six head motion parameters and a constant regressor for each run. The contrast responses were divided into two-time windows at the individual subject level: the visual stimuli lasting 250 ms and the following 1000 ms after visual stimuli disappeared. The analysis was performed: No Go condition vs. baseline condition, Go condition vs. baseline condition, and No Go condition vs. Go condition (intergroup comparisons). A second-order group-level random-effect analysis was then implemented across the maps, using the permutation-based nonparametric method [15] to run 5000 permutations in the DPABI software [16]. We had initially set a primary voxel-level threshold at *p* < 0.05 and a minimum extent of 30 voxels in order to form activation clusters. Brain activation was anatomically labeled according to revised atlas AAL2 [17], which was rendered using the bspmview toolbox (10.5281/zenodo.168074).

## 3. Results

The results have shown that, compared with the control group, the exercisers' brain activation of the frontal and center parietal lobes has been positively enhanced during attentive visual perception (Figure 1, Table 2). In the following time, almost the same brain areas of the exercisers responded stronger in negative inhibition control than the control group (Figure 2, Table 3).

## 4. Discussion

This study surveyed the neurophysiological responses of the frequent jogging group using classic GNG paradigms. The exercise group has shown more robust activation of areas like the putamen, thalamus, lingual, fusiform, PFC, and caudate within the perceptive stage than the control group, whereas during the next inhibitory control stage, most of the areas mentioned above of the exercise group have shown augmented inhibitory response compared to the control group. The enhanced responses involved not only activation but also deactivation. Such effects of the temporal dynamic neural network patterns might closely relate to specific functional plasticity shaped by the regular exercise. The two cognitive benefits of increased attention capacity and inhibitory control are focused on being discussed below.

A recent meta-analysis study has demonstrated that physical exercise training leads to changes in functional activation patterns primarily located in the precuneus and associated with frontoparietal, dorsal attention, and default mode networks [18]. Notably, the long-term exercisers have reshaped regions connected with frontoparietal and dorsal attention networks. Our observation is consistent with the previous results. The increased responses of the visual cue-induced reactivity of the exercise group (Table 3) involved mainly the functional networks such as visual information processing (fusiform, lingual gyrus), motivation, and expectation (prefrontal regions). The lateral temporal lobe, including the middle temporal gyrus, has been suggested to consist of the visual association cortex [19]. The visual association cortex has been recently shown to play a role in forming associative memories [20]. Hence, consistent with previous studies of exercise, brain, attention, learning, and memory areas have been reported for cue reactivity, and associative learning plays a significant role in motion maintenance. The enhanced fMRI BOLD response in the functional areas' dopaminergic neuron activity in regions of the frontal cortex (FC) is postulated to be involved in conditioning for reward expectancy from sensory cues [21, 22].

Additionally, PFC, connecting neuroanatomically with limbic structures, is believed to be more responsible for reward expectancy's emotional and motivational features [23]. As expected, the enhanced activation of PFC in our study suggested that the exercise group is more sensitive and attentive with visual stimuli, and consequently, the motivational networks are overexcited. PFC is considered engaged with memory and reward expectancy by evaluating and integrating sensory input and affective information [24–26], leading to goal-directed action [27]. Hence, our observation supported the hypothesis that the enhanced activation of PFC indicates that the exercise subjects were more sensitive and attentive to the visual stimuli.

During the following inhibition control process (NoGo > Go), the exercise group showed significant deactivation in the left and right thalamus, putamen, caudate, lingual, PFC, and anterior cingulum (Table 3). Almost the same brain areas, which have been involved in overexcitation (more positive) at the perception stage (receiving the visual image), have been switched to more substantial inhibitory control (more negative) for the following decisive process (Go or No Go). Such activity may imply stronger activity of the brain for inhibitory control in the exercise group. Previous literature has shown that inhibitory control is a crucial component common to executive functions [28]. On one side, the development of inhibitory control with the children has a massive impact on their academic achievement [29, 30] and mental health [31]. On the other side, poor inhibitory control predicts risky addictive behaviors. For example, a study of the Internet gaming disorder group has shown more impulsivity and lower activity of the right Secondary Motor Area (SMA)/pre-SMA compared to the control group [32]. Combining both the aspects of the salience of gambling-related cues and response inhibition, using the GNG task, van Holst et al. [33] showed lower activation of the dorsolateral and anterior cingulate cortex during neural inhibition in individuals with gambling disorder. Ding et al. [34] observed both enhanced and reduced responses in different brain areas with the NoGo task. The subjects with Internet game addiction exhibited hyperactivity during No Go trials in the left superior medial frontal gyrus, right anterior cingulate cortex, right superior/middle frontal gyrus, left inferior parietal lobule, and left precentral gyrus, as well as the left precuneus and left cuneus. Meanwhile, several brain regions exhibited decreased activity, including in the bilateral middle temporal gyrus, bilateral inferior temporal gyrus, and right superior parietal lobule. This hypeactivation might be an impairment in turning off the default mode during No Go trials. Based on the inhibitory control impairment of addictive behavior, some literature has reported that exercise can be effective for addiction treatment [35]. Thus, it is essential to understand the details of the temporal neural dynamic patterns involved in the inhibitory control process, indicating the mechanism of neuroplasticity shaped by exercises.

Although this study was to explore the exercise-brain mechanism with fMRI, there are some limitations. Some more specific experiment paradigms, like selective attention with exercise-related images, may help further to analyze the task-specific attention, reward, and task-related cognitive benefits. In the future, a detailed analysis of the GNG behavior data could be looked at, such as correct and incorrect response ratios and the corresponding brain activities. The stimuli can be replaced with sports pictures instead of classic GNG alphabets. Such modification of experiments can help to observe more specific task-related responses. Moreover, the participants of the exercise are recruited from the jogging club. It could be extended to adopt many other exercisers such as football players and basketball players. The average age of the participants in this study was around the fifties. It would be better to categorize young (below 35, the cognitive function not affected with age) or elders (above 60, the cognitive function most probably affected with age) to extend the understanding of the cognitive development benefits with different age groups.

## 5. Conclusion

To conclude, the present GNG study has supported our hypothesis and indicated that the temporal dynamic neural network activities, including the increased positive activation and stronger inhibitory control located in the frontal and parietal lobes, exhibit the cognitive benefits of regular joggers.

## Figures and Tables

**Figure 1:** Full view of the brain response differences between the exercise and control groups with visual stimuli (*t*-value map). The color bar on the right side indicates the brain activity level.

**Figure 2:** Full view of the brain response differences between the exercise and control groups after visual stimuli (*t*-value map). The color bar on the right side indicates the brain activity level.

**Table 1:** Exercise data and EAI scores of the excessive exercise and the control groups.

	Exercise group	Control group	*t*	df	*p*
Times per week	4.14 ± 1.01	1.31 ± 1.09	10.02	53	≤0.001
Hours per time	1.22 ± 0.47	0.63 ± 0.57	4.25	53	≤0.001
Total exercise time	5.11 ± 2.84	1.14 ± 1.13	6.66	53	≤0.001

**Table 2:** The contrast responses to visual stimuli between exercise and control groups.

Labels	Clusters	*t*	MNI		
			*x*	*y*	*z*
Putamen_L	63	2.85	-33	0	3
Putamen_R	96	2.84	27	15	-3
Thalamus_L	668	3.38	0	-27	3
Lingual_L	668	3.14	-24	-48	-3
Fusiform_L	668	3.11	-30	-58	-6
Lingual_R	80	2.57	24	-45	-3
Thalamus_R	65	2.02	9	0	21
PFC_L	660	3.03	-27	45	3
PFC_R	660	2.28	33	36	0
Caudate_L	660	3.27	0	0	9
Caudate_R	660	2.49	24	27	3
PFC_R	36	2.03	-54	21	27

Regions were automatically labeled using the Anatomy Toolbox atlas.*x*,*y*, and*z* = Montreal Neurological Institute (MNI) coordinate in the left-right, anterior-posterior, and inferior-superior dimensions, respectively. Results were filtered with a cluster-forming threshold of*p* < 0.05and a cluster-wise minimum cluster size of*k* ≥ 30.

**Table 3:** The contrast responses with inhibitory control between exercise and control groups.

Labels	Clusters	*t*	MNI		
			*x*	*y*	*z*
Frontal_Sup_R	30	2.40	15	15	51
Temporal_Mid_L	31	-2.32	-60	-54	3
Thalamus_L	2472	-2.54	-6	-15	0
Thalamus_R	2472	-2.52	10	-6	9
Putamen_L	2472	-2.72	-30	6	-6
Putamen_R	2472	-2.92	27	15	-3
Caudate_L	2472	-2.36	-7	9	4
Caudate_R	2472	-2.92	15	34	9
Lingual_L	2472	-3.52	-24	-48	-3
Lingual_R	2472	-2.75	27	-48	-2
PFC_L	2472	-3.02	-27	45	3
PFC_R	2472	-3.06	6	51	1
Cingulum_Ant_L	2472	-2.18	-5	40	8
Cingulum_Ant_R	2472	-2.03	4	42	8

Region labeling and data filtering were the same as in Table 2.

## Data Availability

The fMRI data used to support the findings of this study are available from the corresponding author upon request.
